# Changes in Chinese early adolescents’ group orientation and mental health from before to during the COVID-19 pandemic

**DOI:** 10.3389/fpsyg.2023.1093128

**Published:** 2023-03-03

**Authors:** Xianguo Han, Yanyu Xia, Panpan Yang, Dan Li, Xuechen Ding, Rongwei Zhang, Minghao Zhang

**Affiliations:** ^1^Department of Psychology, Shanghai Normal University, Shanghai, China; ^2^Department of Public Administration, Fujian Provincial Party School of CPC, Fuzhou, China; ^3^Department of Public Administration, Fujian Academy of Governance, Fuzhou, China; ^4^School of Science and Education, Ludong University, Shangdong, China

**Keywords:** COVID-19, group orientation, mental health, rural–urban difference, Chinese early adolescents

## Abstract

Adolescence is a critical period for formulating and developing value orientations. The COVID-19 pandemic has dramatically restricted people’s lives, potentially leading adolescents to reevaluate what they prioritize in life (i.e., their values) and affecting their mental health. Previous studies suggest that Chinese early adolescents’ group orientation is negatively associated with mental health more strongly in rural than in urban, whereas this rural–urban differs may vary after the outbreak of the pandemic. To examine potential changes in group orientation, mental health, and their associations during the pandemic, two cross-sectional surveys of ninth-grade students in the same three school were conducted in rural and urban China in 2019 and 2021. The results showed that compared with students before the pandemic (2019, *N* = 516, 48.8% girls, M_age_ = 14.87 years), students during the pandemic (2021, *N* = 655, 48.1% girls, M_age_ = 14.80 years) displayed lower group orientation such as group responsibility and rule abiding of rural students, and higher loneliness and depressive symptoms. Social equality, group responsibility and rule abiding were all significantly negatively associated with loneliness and depressive symptoms. Those negative associations were stronger in the urban regions than in the rural region. Follow-up invariance analysis revealed that this rural–urban difference in the relations between social equality, group responsibility, and rule abiding and mental health problems was only significant during (and not before) the pandemic. The protective effect of group orientation on mental health seems to be weakened only in rural contexts. The results suggest that significant changes in macrolevel contexts may play an important role in shaping adolescents’ value orientation and mental health.

## 1. Introduction

Since the World Health Organization declared the novel coronavirus disease (COVID-19) a pandemic on 11 March 2020, the surge of infections seriously threatened citizens’ lives and posed a significant challenge to national healthcare systems (Zhang N. et al., 2022). To interrupt the spread of the pandemic, some preventive and suppressive measures have been implemented worldwide, including school closures, social distancing, and masking (Zhang N. et al., 2022). The true extent of the pandemic is not yet known, yet research already suggests that COVID-19 will have a persistent and profound impact on individuals’ mental health and wellbeing, especially for at-risk and vulnerable groups such as children and adolescents, infected and suspected infected individuals, medical frontline workers, home isolators, older adults (65 years and older), chronically ill patients, and disabled persons (Zhang N. et al., 2022). Children and adolescents, in particular, have limited event interpretation skills and coping strategies, which may leave them more vulnerable to psychological health problems during the pandemic (Dalton et al., 2020). Moreover, online teaching and prolonged home isolation have reduced opportunities for interacting with peers and teachers, which may undermine the physical and mental health of children and adolescents (Liu et al., 2021; Lichand et al., 2022). For instance, researchers found that Norwegian adolescents had higher depressive symptoms and lower optimism about their future lives during (relative to before) the pandemic (von Soest et al., 2022).

The COVID-19 pandemic greatly affected people’s lives, potentially leading individuals to reevaluate their views and beliefs regarding what is important (Daniel et al., 2021). Value orientations reflect what people prioritize in life (Schwartz, 1992), and thus form the basis for constructing belief systems on what is right or wrong, good or bad. Adolescents’ value orientations could be directly associated with their mental health: for instance, group orientation has been found to significantly weaken children’s loneliness and depressive symptoms (e.g., Liu et al., 2018). Shifts in the values of early adolescents during the COVID-19 pandemic may have far-reaching consequences for the societal future, particularly those regarding group orientation, which is highly valued in traditional Chinese culture. Early adolescence is a critical time for formulating and developing value orientations, which are susceptible to influence by society, school, family, and peers (Sagiv and Schwartz, 2022). Moreover, as regional culture differs between urban and rural areas in China, the association between group orientation and mental health may vary (Chen et al., 2012; Liu et al., 2018). It will be interesting to investigate how adolescents’ group orientation, mental health, and their associations change in the rural and urban environment during a continuous crisis.

### 1.1. Early adolescents’ group orientation during COVID-19

Group orientation is characterized by concern for group welfare and collective harmony (Chen et al., 2012). Higher group-oriented individuals are more likely to display responsiveness and respect, especially when expressing their own views and feelings, which is extremely important to maintain group functioning and positive social relationships (Kitayama et al., 2010). As a core component of the self, value orientations have great stability through life but are also adaptive and may be altered by the external environment, especially for adolescents (Alvarez et al., 2021; Daniel et al., 2021). Early adolescence is an important period in the development of identity and autonomy (Kroger et al., 2010) and the emergence of mental health problems (Kessler et al., 2005). As their need for autonomy and independence awakens, adolescents are generally more open to change than adults, and place a higher value on hedonism and stimulation, as well as personal success, achievement, and power (Alvarez et al., 2021). However, the value orientations of early adolescents are susceptible to influence by surroundings, and could thus be altered by life adversities such as the spread of major infectious diseases (e.g., COVID-19).

In most studies of changes in personal values during the pandemic, researchers have used of 10 basic individual values identified by Schwartz (1992). In the Schwartz value theory, values are structured on a circular continuum according to their expressed motivations. Adjacent values express compatible motivations, while opposing values express conflicting motivations, categorized by two pairs of higher-order dimensions (e.g., Daniel et al., 2021; Sagiv and Schwartz, 2022). On the one hand, the openness to change vs. conservation dimension captures the conflict between the motivation to promote creativity, independence, novelty, and excitement expressed by self-direction, stimulation, and hedonism values. On the other hand, motivation to maintain order and safety and resistance to change is expressed by conformity, tradition, and security values. Similarly, the self-transcendence vs. self-enhancement dimension captures the conflict between the motivation to promote concern for the welfare of others, as expressed by universalism and benevolence values; the motivation to promote self-interest, success, and dominance is expressed by power and achievement values. Previous studies have found that major existential threats can change an individual’s value orientation. For example, in the aftermath of the 2008 financial crisis (Sortheix et al., 2019) and exposure to war (Daniel et al., 2013), early adolescents’ conservation values became more important, while motivationally opposing values, including self-direction, stimulation, and hedonism, weakened. According to evolutionary theory, the collective behavioral reactions to major infectious diseases could lead to adaptive change in an individual’s value orientations (Thornhill and Fincher, 2014). To reduce disease spread during a disaster, behavioral avoidance systems (e.g., decreased out-group contact) and conservation values may be activated (Woltin and Bardi, 2018). Previous studies have also documented systematic population-wide changes in personal values during the COVID-19 pandemic. Some longitudinal studies have reported that conservation values have strengthened, while self-transcendence values have weakened during the pandemic (Daniel et al., 2021; Yu et al., 2022). According to the terror management theory (Greenberg et al., 1986), there are conflicting predictions of changes in self-transcendence. Increased mortality is likely to increase the willingness to defend one’s own worldview (Burke et al., 2013), which could decrease the value of the universalism aspect (concern for welfare of all) of self-transcendence (Courtney et al., 2020). However, other studies found that increased mortality salience would provoke enhanced associations with close others after major existential threats (Mikulincer et al., 2003), thereby increasing the importance of the benevolence aspect (concern for welfare of close others) of self-transcendence. Daniel et al. (2021) explored these effects in Australian adults and revealed that the outbreak of the pandemic was initially followed by declining concern for distant others, society, and nature; later, connections with close others began falling too. Over time, the decreased importance of self-transcendence values was more likely in individuals with high levels of worry about the pandemic than those with medium or low levels of worry.

Notwithstanding the robustness of the evidence produced under the theory identified by Schwartz (1992), thus far, relevant research on the pandemic has mostly focused on values in adults and adolescents (Russo et al., 2022; Sagiv and Schwartz, 2022), with a paucity of evidence on the younger population, namely early adolescents. Therefore, this study will explore the change of group orientation from before to during the pandemic in Chinese early adolescents.

### 1.2. Group orientation and mental health in rural and urban contexts

China is considered a collectivist society, with Confucianism as the predominant ideology guiding people’s lives (Ho, 1986; Yang, 1986). Confucianism requires that people restrain their behaviors and emotions to maintain positive social relationships and group harmony (i.e., Chen et al., 2012). Chinese society encourages concern for group functioning and prioritizing collective welfare over one’s own benefit, especially amid the emerging conflict between individual and collective interests (Chen, 2012). Therefore, adolescents who display self-control and value group functioning are more likely to be appreciated by parents, educators, and peers. According to Lu (2006), group orientation creates a “cultural fit” with the social expectations of China’s collectivist culture. It has also been shown to be positively associated with psychosocial adjustment: for instance, adolescents who focus more on group orientation have greater social competence and higher self-esteem, while also experiencing less loneliness and depressive symptoms (Chen et al., 2012; Liu et al., 2018; Wang et al., 2018; Tan et al., 2021).

Studies on how context affects the relationship between value orientations and mental health suggest that the same value orientation may relate positively or negatively to mental health, depending on the social context (Sagiv and Schwartz, 2022). Value orientation may create or enhance positive associations with mental health if pursuing the value helps the individual overcome contextual obstacles. Before the pandemic, unprecedented market-oriented reforms and increasing urbanization dramatically changed Chinese social circumstances (Chen et al., 2005, 2012). Notably, individualism is on the rise, while collectivism is declining (Cai et al., 2020). Self-orientation, which emphasizes personal competition and independence, is increasingly accepted, particularly by the young urban generations (Chen et al., 2005, 2021; Liu et al., 2018). For example, a study of 6th to 12th grade Chinese students revealed that individualistic orientation positively contributed to adolescents’ perceived self-worth (Tan et al., 2021). However, the large-scale market-oriented reform and urbanization in China has been largely limited to urban centers and cities. In rural regions, the group orientation traditionally endorsed by Confucian ideologies is still more likely to prevail (Liu et al., 2018; Yue et al., 2020). It has been found, for example, that compared to their urban peers, rural adolescents who emphasize group orientation will receive more social reinforcement and experience fewer emotional functioning problems (Chen et al., 2012; Liu et al., 2018).

It is noteworthy that although individuality, independence, and autonomy increase with rapid urbanization and individualization in early adolescents, they do not necessarily reduce their need for social relationships and a sense of belonging (Kagitcibasi and Ataca, 2005). Group orientation, such as social harmony and obedience, persists, and even strengthens, in modern Chinese society (Zeng and Greenfield, 2015; Zhou et al., 2018). Chen et al. (2012) found that urban youth’s self- and group-orientation values become more coexisted and integrated in China. A recent three-year longitudinal study examined the developmental trajectories of value orientations across early adolescents. The study found that early adolescents’ self- and group-orientation values increased in linear trajectories (Chen et al., 2018). Li et al. (2018) found that group orientation (i.e., social equality, group responsibility, and rule-abiding) was higher in urban cities than rural areas, and that the alleviative effect of group orientation on depressive symptoms did not vary with urbanization. Therefore, the relationships between group orientation and mental health in Chinese early adolescents are not inevitably stronger in rural than in urban areas, depending on various situational factors.

Major life events may cause substantial changes in people’s values and their relationship with mental health. Whether new variations in rural–urban differences have emerged following the COVID-19 outbreak in the relationship between Chinese early adolescents’ group orientation and mental health remains to be seen. China was the first country to adopt strict measures against the spread of the virus, such as school closures, physical distancing, and restrictions on recreational activities (Qi et al., 2022). These measures kept infections and deaths to very low levels, while also negatively impacted on the economy, employment, and public health (Zhang Q. et al., 2022). Researchers have suggested that the prevalence of mental health problems (e.g., depression and anxiety symptoms) in children and adolescents has increased considerably during COVID-19 (e.g., Racine et al., 2021).

There is also mixed evidence on rural–urban differences in the relationship between group orientation and mental health after the outbreak of the pandemic. Some studies have found that, compared to cities, the protective effect of group orientation on mental health seems to enhanced in rural contexts during the pandemic. For example, rural migrant children and left-behind children appeared to have higher psychological wellbeing than urban children during the initial phase of the COVID-19 outbreak in China (e.g., Zhang R. et al., 2022). Compared with United States and Japanese participants, Chinese participants had a stronger link between societal considerations and higher acceptance of society-level preventive measures (e.g., school closure) during the COVID-19 pandemic (Zhu et al., 2021). Zhu et al. (2020) argued that the learning style that adolescents adopt to cope with uncertainty threats in different cultural contexts may have profound psychological implications. Compared with adolescents in individualistic cultures who use an individual learning style (i.e., a free, independent search for innovative solutions) to enhance their sense of control, adolescents in collectivistic cultures who adopt a social learning style (i.e., copying existing solutions with deference and conformity) are more likely to benefit from those reconcile measures during the COVID-19 pandemic.

However, depending on the continuation of new life conditions, the longevity of changes in value may affect their relationship with mental health. Previous studies have pointed out that value orientations have returned to normal, such as openness to change in Australia in late 2020 (Daniel et al., 2021). Approximately 2 years following the outbreak, China entered a relatively stable stage of prevention and control of COVID-19 with low contagiousness and low mortality. Adolescents’ fear and anxiety have alleviated, and the need for self-direction has increased consistently (e.g., Yu et al., 2022). While urban residents recovered quickly when virus transmission was effectively contained, the impact of the pandemic on rural regions remains unresolved, if not intensified (Shen et al., 2021). This suggests that when the virus spread is effectively contained, the return of value orientation among early adolescents in rural areas may be somewhat higher than in urban areas. Relatively low socioeconomic status, unfavorable learning environment, and the coexistence contradiction between excessive supervision and frequent violations of pandemic prevention measures may be important factors hindering group orientation reacquisition. In this study, we explore whether there are new patterns of change in early adolescents’ group orientation in relation to mental health that emerged among rural and urban samples from before to during the pandemic.

### 1.3. The present study

The COVID-19 pandemic greatly affected adolescents’ lives, which may have impacted on their views and beliefs on what is important (i.e., their values; Daniel et al., 2021). The primary purpose of this study is to examine the relationships between group orientation and mental health in Chinese early adolescents before and during the COVID-19 pandemic. The study used two samples of ninth-grade students from three regular public junior high schools in rural and urban regions: the first sample was surveyed in 2019 and the second in 2021. The ninth-grade is a critical period in adolescents’ formulation and development of their values and beliefs (Li et al., 2018; Wang et al., 2018). Additionally, Chinese entrance exams for high school place significant pressure on ninth graders, even during COVID-19 quarantine. Chinese adolescents’ academic success or failure can have a ripple effect on their self-perception (e.g., self-esteem) and mental health problems including loneliness and depressive symptoms (e.g., Liu et al., 2018; Tan et al., 2021).

As Heim et al. (2019) contends, to produce meaningful findings on correlations between personal value orientations and self-reported symptoms of psychopathology, the cultural context must be considered. Dramatic social changes in China have resulted co-existence between modern and traditional values; the ideal and the secular; collectivism and individualism. To reveal changes in adolescents’ values, Wang et al. (2018) developed the Adolescent Values Questionnaire (AVQ) based on contemporary China. This questionnaire has demonstrated high levels of reliability and validity in assessing the value orientations of Chinese adolescents (Li et al., 2018; Wang et al., 2018). In the present study, we chose social equality, group responsibility, and rule-abiding as indicators to reflect three aspects of group orientation. Social equality captures the approval of social norms and justice, concerns about social status, and respect for human rights. Group responsibility embodies concerns and preferences for group interests. Valuing group responsibility does not mean that individuals must sacrifice their independence; rather, they express the desire to integrate, belong, and grow together with the group. Rule-abiding captures an individual’s adherence to social rules, laws, traditions, and customs, which is consistent with the concern for self-discipline and obedience advocated by Confucianism and Taoism in traditional Chinese culture. Previous studies have found that social equality, group responsibility and rule abiding were significantly negatively associated with mental health problems such as depressive symptoms (Li et al., 2018). By comparing the AVQ with Schwartz’s (2005) theory of the structure of values, Wang et al. (2018) suggested that social equality is related to the universalism aspect of self-transcendence, rule-abiding is related to conservation value, and group responsibility is related to social-focused values that are directed toward the interests of the closer social network or society at large. Regarding youth mental health, loneliness and depressive symptoms are considered important indicators in the time of COVID-19 (e.g., Brooks et al., 2020). Moreover, previous studies have found that gender and parental education level may be related to group orientation and mental health (Liu et al., 2018; Zhao et al., 2022). Accordingly, we added both as control variables.

The current study is the first application of the Adolescent Values Questionnaire (AVQ) in contemporary China to examine the changes in value orientation and mental health problems of early adolescents before and during the pandemic. Based on previous theoretical and empirical studies (e.g., Daniel et al., 2021; Yu et al., 2022), we hypothesized that following the outbreak of COVID-19, Chinese early adolescents’ social equality and group responsibility decrease, and rule abiding increase. In addition, based on the literature on rural–urban differences in China (e.g., Liu et al., 2018; Zhu et al., 2020, 2021), we expected the relationships between group orientation particularly group responsibility and mental health to be stronger in rural contexts than in urban ones.

## 2. Materials and methods

### 2.1. Participants

Of the three schools selected for the cross-sectional surveys, two were located in urban areas (Yantai, Shandong Province, and Shanghai) and one was in a rural area (Anyang, Henan Province). The sample for the first survey (November 2019, before the pandemic) comprised 516 ninth-grade students (48.8% girls, 69.4% urban residents, M_age_ = 14.87 years, SD = 0.54). Regarding parents’ education level, 66.9% of fathers and 73.7% of mothers had not progressed beyond junior high school, 28.2% of fathers and 21.1% of mothers had achieved a senior high school degree, and the remainder had achieved a college degree or completed higher education. Two years later(November 2021), the second survey was conducted with a new sample of 655 ninth-grade students (48.1% girls, 56.8% urban residents, M_age_ = 14.80 years, SD = 0.57) from the same three schools. As regards parents’ education level, 59.9% of fathers and 64.8% of mothers had not progressed beyond junior high school, 25.8% of fathers and 21.9% of mothers had achieved a senior high school degree, and the remainder had achieved a college degree or completed higher education. The rural and urban adolescents did not differ on age [*t*(1125) = 1.89, *p* > 0.05] or gender [*χ*^2^(1) = 0.07, *p* > 0.05], but urban fathers [*χ*^2^(2) = 141.66, *p* < 0.001] and mothers [*χ*^2^(2) = 105.77, *p* < 0.001] were more likely than their rural equivalents to have achieved a senior high school degree or completed higher education. The parental educational levels in this sample were similar to those reported for the general population in the regions (Bureau of Statistics of Anyang, 2021; Bureau of Statistics of Shanghai, 2021; Bureau of Statistics of Yantai, 2021). Most participants in both samples were of Han nationality, which is the predominant ethnic group in China (over 90% of the population). Almost all participants were of native residence (over 80% of the population). Preliminary analyses indicated no significant differences between Shanghai and Yantai in the relations between group orientation and mental health problems. Basic characteristics of socioeconomic indicators are presented in Table 1.

**Table 1:** Basic characteristics of socioeconomic indicators.

Variables		Before the pandemic				During the pandemic			
		Urban		Rural		Urban		Rural	
		*N*	%	*N*	%	*N*	%	*N*	%
Full sample		358	69.4	158	31.6	372	56.8	283	43.2
**Gender**									
Girl	166	46.4	86	54.4	184	49.5	131	46.3
Boy	191	54.6	72	45.6	182	51.5	152	54.7
**Father education**									
Junior high school and below	189	58.5	122	85.9	144	41.7	225	83.0
Senior high school	112	34.7	19	13.4	114	33.0	45	16.6
College and above	22	6.8	1	0.7	87	25.3	1	0.4
**Mother education**									
Junior high school and below	216	66.1	126	92.0	173	49.9	226	84.0
Senior high school	88	26.9	10	7.3	97	28.0	38	14.1
College and above	23	7.0	1	0.7	77	22.1	5	1.9
**Native residence**									
Yes	274	80.8	137	99.3	288	81.4	274	98.9
No	65	19.2	1	0.7	66	18.6	3	1.1

### 2.2. Measures

#### 2.2.1. Group orientation

Group orientation of early adolescents was assessed using the Adolescent Values Questionnaire developed by Wang et al. (2018). The original instrument comprises 46 items across eight dimensions: social equality, group responsibility, rule abiding, family wellbeing, friendship, self-improvement, fashion, and personal happiness. Each item describes a person’s view or belief, and participants report the extent to which that view/belief matches their own, responding on a five-point scale from 1 (“not like me at all”) to 5 (“very much like me”). Previous studies have shown that this scale has high levels of reliability and validity in the Chinese cultural context (Li et al., 2018; Wang et al., 2018). As this study focused more on the early adolescents’ concern for group welfare and collective harmony than the concern for self- or close others’ interests, according to the recommendations of Wang et al. (2018), the following were used as indicators of group orientation: social equality (six items, e.g., “He/she believes that all people are equal, regardless of race, gender, social status, etc.”); group responsibility (seven items, e.g., “He/she believes that people can forsake their own interests to promote group functioning”); rule abiding (five items, e.g., “He/she believes that everyone has to abide by discipline and rules”). Standardized loadings ranged from 0.468 to 0.836, and the three-factor model had acceptable goodness of fit for the before- and during-pandemic groups: *χ^2^*(129) = 308.486 and 376.825, comparative fit index (CFI) = 0.929 and 0.940, root mean squared error of approximation (RMSEA) = 0.052 and 0.054, standardized root mean square residual (SRMR) = 0.044 and 0.039, respectively. The Cronbach’s alpha coefficients for social equality, group responsibility and rule abiding before and during the pandemic were 0.826, 0.849, 0.836 and 0.885, 0.872, 0.876, respectively.

#### 2.2.2. Loneliness

Early adolescents’ loneliness was assessed using Illinois Loneliness Scale, a self-report measure adapted from Asher et al. (1984). The measure comprises 16 statements describing loneliness (e.g., “I have nobody to talk to”; “I feel lonely”), and participants respond by indicating the extent to which each statement applies to them. Responses are given on a 5-point scale, ranging from 1 (“not at all true”) to 5 (“always true”). Previous studies have shown that this scale has high levels of reliability and validity in a Chinese cultural context (e.g., Liu et al., 2021). Standardized loadings ranged from 0.376 to 0.821, and the five-factor model had acceptable goodness of fit for the before- and during-pandemic groups: *χ^2^*(92) = 226.93 and 300.50, CFI = 0.942 and 0.940, RMSEA = 0.053 and 0.059, SRMR = 0.047 and 0.057, respectively. The Cronbach’s alpha coefficients for loneliness before and during the pandemic were 0.862 and 0.877, respectively.

#### 2.2.3. Depressive symptoms

Depressive symptoms in early adolescents were measured through the Childhood Depression Inventory, developed by Kovacs (1985) and revised by Chen et al. (2005). The inventory comprises 14 items covering a wide range of typical depressive symptoms, such as sleep disorders, loss of appetite, and suicidal ideation. Each item is answered on a three-point scale and the scores for reverse questions are transformed to obtain the mean score. A higher score indicates stronger depressive symptoms. The inventory has shown relatively high reliability and validity for a Chinese adolescent sample (Liu et al., 2014). Standardized loadings ranged from 0.371 to 0.729, and the one-factor model had acceptable goodness of fit for the before- and during-pandemic groups: *χ^2^*(73) = 175.56 and 187.12, CFI = 0.926 and 0.944, RMSEA = 0.052 and 0.049, SRMR = 0.043 and 0.039, respectively. The Cronbach’s alpha coefficients for depressive symptoms before and during the pandemic were 0.856 and 0.867, respectively.

### 2.3. Procedure

After obtaining the consent of the school, data collection was conducted in 2019.11 (before the pandemic) and 2021.11 (about 2 years after the outbreak of the pandemic). The procedure was the same in the urban and rural groups. All researchers involved in collecting data were Ph.D. or master’s students majoring in developmental and educational psychology. Prior to data collection, they underwent training in psychological assessment. When administering the questionnaire survey, the researchers explained to participating students and their parents/legal guardians the study’s purpose, that responses would remain confidential, and that participation was entirely voluntary. In the study, participants completed self-report measures of group orientation, loneliness, and depressive symptoms. It took approximately 30 to 45 min to complete the measures. All participating students and their parents (or legal guardians) signed the informed consent form before the survey.

### 2.4. Data analysis

We first examined measurement invariance for group orientation, loneliness, and depressive symptoms. The latent constructs of social equality, group responsibility and rule abiding as well as loneliness and depressive symptoms were formed based on the corresponding items. Then, we tested the main effect of group orientation on loneliness and depressive symptoms through structural equation modeling. Finally, a set of multigroup invariance tests were conducted to assess overall differences across rural–urban group and rural–urban group interactions with before-during pandemic in the relations. A significant difference in χ^2^ between the constrained model (all the paths were set equal across groups) and the unconstrained model (all the paths were freed across groups), which calculated by Wald Chi-square test, indicated the path coefficients in the relations could not be considered equivalent between the groups. When overall group differences are found, the sources of difference will be investigated through follow-up invariance tests on specific path coefficients across rural–urban group, constraining individual relations between group orientation and mental health problems. In structural equation modeling and multigroup invariance tests, we controlled for adolescent’s gender and parental education level (the mean of mother and father educational levels). The analyses were conducted in Mplus 7.4 (Muthén and Muthén, 2012).

Overall model fit was evaluated by four indices: chi-square goodness-of-fit statistic, CFI, RMSEA, and SRMR. The criteria for acceptable model fit were CFI ≥ 0.90, RMSEA ≤ 0.06, and SRMR ≤ 0.08 (Hu and Bentler, 1999). We also reported 95% bias-corrected confidence intervals (95% CI), with significance denoted by the 95% CI not including zero (MacKinnon et al., 2004).

## 3. Results

### 3.1. Measurement invariance

We tested measurement invariance of group orientation, loneliness, and depressive symptoms by fitting and comparing a series of sequentially more constrained models. The aim was to verify that the factor loadings and intercepts for indicators were invariant across rural–urban group, before-during pandemic group, and gender. Measurement invariance was tested by using chi-square values and the changes in the value of CFI, RMSEA, and SRMR (Chen, 2007). Significant chi-square test results suggest potential heterogeneity of the model across groups, while small changes in SRMR, CFI, and RMSEA suggest model invariance (Chen, 2007). Because of Chi-square tests are sensitive to sample size and may incorrectly reject measurement invariance, we further applied the change criteria of CFI, RMSEA and SRMR to ascertain measurement invariance in cases of significant chi-square test results. We examined the invariance of loadings, intercepts, and means of the model. Specifically, for testing loading invariance, ΔCFI ≥ 0.010, ΔRMSEA ≥ 0.015, or ΔSRMR ≥ 0.030 indicated non-invariance; for testing intercept invariance, ΔCFI ≥ 0.010, ΔRMSEA ≥ 0.015, or ΔSRMR ≥ 0.010 indicated non-invariance (Chen, 2007). As shown in Table 2, the results indicate that factor loadings and (partial) intercepts invariance was established for group orientation, loneliness, and depressive symptoms.

**Table 2:** Fit statistics for measurement model and tests of measurement invariance.

Model	Model χ^2^ (*df*)	Δχ^2^(*df*), *p*	RMSEA	CFI	SRMR	ΔRMSEA	ΔCFI	ΔSRMR
**Group orientation**								
**Rural–urban group**								
Configural	665.900(258)		0.052	0.941	0.040			
Loadings	694.490(273)	25.62(15), <0.05	0.051	0.939	0.049	−0.001	−0.002	0.009
Intercepts	730.310(288)	34.62(15), <0.01	0.051	0.936	0.050	0.000	−0.003	0.001
**Before-during pandemic**								
Configural	685.910(258)		0.053	0.936	0.041			
Loadings	703.610(273)	13.74(15), >0.05	0.052	0.935	0.047	−0.001	−0.001	0.006
Intercepts	735.100(288)	27.26(15), <0.05	0.051	0.933	0.049	−0.001	−0.002	0.002
**Gender**								
Configural	653.26(258)		0.051	0.941	0.039			
Loadings	676.25(273)	19.59(15), >0.05	0.050	0.940	0.049	−0.001	−0.001	0.010
Intercepts	710.87(288)	33.19(15), <0.01	0.050	0.937	0.053	0.000	−0.003	0.004
**Loneliness**								
**Rural–urban group**								
Configural	497.31(184)		0.054	0.947	0.050			
Loadings	521.65(199)	24.29(15), >0.05	0.053	0.945	0.059	−0.001	−0.002	0.009
Intercepts	602.65(214)	93.57(15), <0.001	0.056	0.934	0.059	0.003	−0.011	0.000
Intercepts_m	581.18(213)	69.04(14), <0.001	0.054	0.937	0.059	0.001	−0.008	0.000
**Before-during pandemic**								
Configural	528.83(184)		0.057	0.940	0.053			
Loadings	548.34(199)	19.97(15), >0.05	0.055	0.940	0.058	−0.002	0.000	0.005
Intercepts	581.22(214)	29.88(15), <0.05	0.054	0.937	0.057	−0.001	−0.003	−0.001
**Gender**								
Configural	519.19(184)		0.056	0.940	0.053			
Loadings	537.00(199)	18.46(15), >0.05	0.054	0.940	0.058	−0.002	0.000	0.005
Intercepts	631.21(214)	114.18(15), <0.001	0.058	0.926	0.061	0.004	−0.014	0.003
Intercepts_m	599.65(212)	78.11(13), <0.001	0.056	0.931	0.061	0.002	−0.009	0.003
**Depressive symptoms**								
**Rural–urban group**								
Configural	353.72(146)		0.049	0.940	0.040			
Loadings	370.24(159)	17.80(13), >0.05	0.048	0.939	0.048	−0.001	−0.001	0.008
Intercepts	416.30(172)	49.12(13), <0.001	0.049	0.929	0.049	0.001	−0.010	0.001
**Before-during pandemic**								
Configural	362.66(146)		0.050	0.937	0.041			
Loadings	366.93(159)	6.72(13), >0.05	0.047	0.939	0.045	−0.003	0.002	0.004
Intercepts	408.11(172)	43.50(13), <0.001	0.048	0.931	0.047	0.001	−0.008	0.002
**Gender**								
Configural	408.62(146)		0.056	0.923	0.044			
Loadings	453.79(159)	44.23(13), <0.001	0.057	0.913	0.067	0.001	−0.010	0.023
Intercepts	510.96(172)	60.52(13), <0.001	0.058	0.900	0.075	0.001	−0.013	0.008
Intercepts_m	483.48(171)	28.97(12), <0.001	0.056	0.908	0.074	−0.001	−0.005	0.007

Configural, testing whether the factor structure is the same across groups; Loadings, testing whether the factor loadings (from items to constructs and from constructs to higher-order constructs) are similar across groups; Intercepts, testing whether model intercepts are also equivalent across groups; Intercepts_m, Intercepts invariance model modified.

### 3.2. Descriptive data

No item has more than 2.39% missingness. Little’s MCAR test (Rubin, 1976) showed that the data were missing completely at random [*χ*^2^(60) = 76.85, *p* > 0.05]. As suggested by other researchers (e.g., Graham, 2009), we used full information maximum likelihood estimation to handle missing data.

A multivariate analysis of variance was conducted to examine gender, before-during pandemic, and rural–urban group on the variables. The results showed that the main effects of rural–urban group [*Wilks’ λ* = 0.945, *F*(5, 1,149) = 13.37, *p* < 0.001, $\eta^{2}$ = 0.055], before-during pandemic group [*Wilks’ λ* = 0.976, *F*(5, 1,149) = 5.71, *p* < 0.001, $\eta^{2}$ = 0.024] and gender [*Wilks’ λ* = 0.944, *F*(5, 1,149) = 13.52, *p* < 0.001, $\eta^{2}$ = 0.056] were all significant. There was a significant interaction effect of rural–urban group and before-during pandemic group [*Wilks’ λ* = 0.990, *F*(5, 1,149) = 2.24, *p* < 0.05, $\eta^{2}$ = 0.010], and other interaction effects were all no significant.

Follow-up univariate analyses revealed that social equality [*F*(1, 1,153) = 21.28, *p* < 0.001, $\eta^{2}$ = 0.018], group responsibility [*F*(1, 1,153) = 12.72, *p* < 0.001, $\eta^{2}$ = 0.011] and rule abiding [*F*(1, 1,153) = 16.32, *p* < 0.001, $\eta^{2}$ = 0.014] were significantly higher, loneliness [*F*(1, 1,153) = 9.00, *p* < 0.01, $\eta^{2}$ = 0.008] and depressive symptoms [*F*(1, 1,153) = 12.86, *p* < 0.001, $\eta^{2}$ = 0.011] were significantly lower before than during the pandemic. Social equality [*F*(1, 1,153) = 15.12, *p* < 0.001, $\eta^{2}$ = 0.011], group responsibility [*F*(1, 1,153) = 12.39, *p* < 0.001, $\eta^{2}$ = 0.011] and rule abiding [*F*(1, 1,153) = 48.10, *p* < 0.001, $\eta^{2}$ = 0.040] were significant higher, loneliness was significantly lower [*F*(1, 1,153) = 4.85, *p* < 0.05, $\eta^{2}$ = 0.004] in the urban regions than in the rural region. Girls reported greater social equality [*F*(1, 1,153) = 17.65, *p* < 0.001, $\eta^{2}$ = 0.015] and rule abiding [*F*(1, 1,153) = 10.67, *p* < 0.001, $\eta^{2}$ = 0.009], loneliness [*F*(1, 1,153) = 9.23, *p* < 0.01, $\eta^{2}$ = 0.008] and depressive symptoms [*F*(1, 1,153) = 21.32, *p* < 0.001, $\eta^{2}$ = 0.018] than did boys. In rural, students reported greater group responsibility and rule abiding before than during the pandemic; these effects were not evident in urban. The means and standard deviations of group orientation and mental health problems are presented in Table 3.

**Table 3:** Means and standard deviations of group orientation and mental health problems(M ± SD).

Variables	Urban region				Rural region			
	Before the pandemic		During the pandemic		Before the pandemic		During the pandemic	
	Girl	Boy	Girl	Boy	Girl	Boy	Girl	Boy
Social equality	4.53 ± 0.57	4.37 ± 0.65	4.45 ± 0.68	4.19 ± 0.86	4.48 ± 0.53	4.24 ± 0.7	4.12 ± 0.75	4.03 ± 0.84
Group responsibility	4.03 ± 0.71	3.94 ± 0.74	3.96 ± 0.77	3.97 ± 0.84	3.98 ± 0.68	3.95 ± 0.69	3.60 ± 0.70	3.71 ± 0.77
Rule abiding	4.47 ± 0.66	4.31 ± 0.70	4.40 ± 0.69	4.22 ± 0.85	4.31 ± 0.63	4.07 ± 0.80	3.91 ± 0.80	3.84 ± 0.89
Loneliness	2.06 ± 0.73	2.00 ± 0.64	2.19 ± 0.71	2.00 ± 0.74	2.11 ± 0.64	2.01 ± 0.52	2.34 ± 0.66	2.17 ± 0.73
Depressive symptoms	1.55 ± 0.39	1.40 ± 0.33	1.60 ± 0.38	1.46 ± 0.34	1.44 ± 0.31	1.43 ± 0.27	1.59 ± 0.37	1.49 ± 0.36

As shown in Table 4, Pearson’s correlation analysis indicated that, for urban adolescents, social equality, group responsibility and rule abiding were significantly negatively associated with loneliness and depressive symptoms before to during the pandemic. For rural adolescents, before the pandemic, social equality, group responsibility and rule abiding were significantly negatively associated with loneliness, however, during the pandemic, only group responsibility was significantly negatively associated with depressive symptoms. In addition, we also found parental education level and adolescent’s gender were both negatively correlated with loneliness and depressive symptoms, while parental education level was significantly positively associated with group orientation. Therefore, we controlled for the influence of parental education level and adolescent’s gender in the subsequent analyses.

**Table 4:** Correlations of study variables in urban and rural groups before and during the pandemic.

Variables	1	2	3	4	5	6	7
**Before the pandemic**							
1. Social equality	1.00	0.73^***^	0.73^***^	−0.35^***^	−0.24^***^	0.19^***^	−0.13^*^
2. Group responsibility	0.65^***^	1.00	0.67^***^	−0.42^***^	−0.25^***^	0.25^***^	−0.06
3. Rule abiding	0.74^***^	0.71^***^	1.00	−0.36^***^	−0.27^***^	0.13^*^	−0.12^*^
4. Loneliness	−0.29^***^	−0.36^***^	−0.32^***^	1.00	0.63^***^	−0.13^*^	−0.04
5. Depressive symptoms	−0.21^**^	−0.29^***^	−0.27^***^	0.61^***^	1.00	−0.07	−0.21^***^
6. Parental education	0.02	0.02	−0.02	−0.16	0.03	1.00	−0.08
7. Gender	−0.19^*^	−0.03	−0.15	−0.08	−0.02	0.002	1.00
**During the pandemic**							
1. Social equality	1.00	0.77^***^	0.82^***^	−0.32^***^	−0.26^***^	0.13^*^	−0.17^**^
2. Group responsibility	0.75^***^	1.00	0.77^***^	−0.47^***^	−0.40^***^	0.10	0.01
3. Rule abiding	0.76^***^	0.71^***^	1.00	−0.35^***^	−0.33^***^	0.14^*^	−0.11^*^
4. Loneliness	−0.16^**^	−0.29^***^	−0.13^*^	1.00	0.62^***^	−0.11^*^	−0.13^*^
5. Depressive symptoms	−0.07	−0.14^*^	−0.08	0.54^***^	1.00	−0.001	−0.19^***^
6. Parental education	0.01	−0.001	0.02	−0.06	−0.09	1.00	−0.06
7. Gender	−0.06	0.07	−0.04	−0.12^*^	0.14^*^	0.09	1.00

Above the diagonal: correlations for urban adolescents; underneath the diagonal: correlations for rural adolescents. Gender (0 = girl, 1 = boy). ^*^p < 0.05, ^**^p < 0.01, ^***^p < 0.001.

### 3.3. Multigroup analysis of the influence of group orientation on mental health problems

We conducted structural equation modeling to test the main effect of group orientation on mental health problems, controlling for adolescent’s gender and parental education. All model of social equality, group responsibility and rule abiding on mental health problems fitted the data well. The results showed that social equality, group responsibility and rule abiding were significantly negatively associated with loneliness (*β =* −0.40 to −0.30, *p*s < 0.001) and depressive symptoms (*β =* −0.35 to −0.28, *p*s < 0.001). Main effect of group orientations on mental health problems are presented in Table 5.

**Table 5:** Main effect of group orientations on mental health problems.

					Goodness−of−fit				
Path	*β*	*SE*	*t*	95% CI	*χ^2^*	*df*	RMSEA	CFI	SRMR
SE on LN	−0.30	0.04	−7.96^***^	−0.37, −0.22	1649.75	615	0.038	0.926	0.052
SE on DS	−0.28	0.04	−7.39^***^	−0.36, −0.21					
GR on LN	−0.40	0.04	−11.07^***^	−0.47, −0.33	1830.00	660	0.039	0.919	0.056
GR on DS	−0.35	0.04	−9.95^***^	−0.41, −0.28					
RA on LN	−0.32	0.04	−8.70^***^	−0.39, −0.25	1689.14	589	0.040	0.920	0.054
RA on DS	−0.31	0.04	−8.41^***^	−0.38, −0.24					

LN, Loneliness; DS, Depressive symptoms; SE, Social equality; GR, Group responsibility; RA, Rule abiding. ^*^p < 0.05, ^**^p < 0.01, ^***^p < 0.001.

Next, we conducted a set of multigroup invariance tests to examine the associations between group orientation and mental health, controlling for adolescent’s gender and parental education. The model of each aspect of group orientation and mental health problems, in which all paths were allowed to vary across rural–urban group, had acceptable goodness of fit (*χ*^2^/*df* = 1.90 to 2.01, RMSEA < 0.042, CFI > 0.915, SRMR < 0.059). The Wald chi-square test indicated there were significant differences in the relations between group orientation and mental health problems across rural–urban group overall [social equality: *χ*^2^(2) = 11.41, *p* < 0.01; group responsibility: *χ*^2^(2) = 7.79, *p* < 0.05; rule abiding: *χ*^2^(2) = 9.54, *p* < 0.01]. Follow-up invariance tests showed that social equality, group responsibility and rule abiding were negatively associated with loneliness and depressive symptoms more strongly in urban than in rural [*χ*^2^(1) = 4.94 to 14.46, *p*s < 0.05]. The results of the tests and the effects of group orientation on mental health problems across rural–urban group are presented in Table 6.

**Table 6:** Multigroup invariance of group orientation on mental health problems across rural–urban group.

	Rural				Urban				
Path	*β*	*SE*	*t*	95%CI	*β*	*SE*	*t*	95%CI	*χ^2^*(1)
**SE on MHP**									
SE on LN	−0.19	0.06	−3.01^**^	−0.32, −0.07	−0.37	0.05	−8.19^***^	−0.46, −0.28	12.91^***^
SE on DS	−0.18	0.07	−2.49^*^	−0.32, −0.04	−0.36	0.04	−8.45^***^	−0.44, −0.28	8.89^**^
**GR on MHP**									
GR on LN	−0.28	0.06	−4.60^***^	−0.40, −0.16	−0.47	0.05	−10.38^***^	−0.55, −0.38	7.08^**^
GR on DS	−0.23	0.07	−3.42^***^	−0.36, −0.10	−0.42	0.04	−10.67^***^	−0.50, −0.34	6.44^*^
**RA on MHP**									
RA on LN	−0.21	0.06	−3.33^***^	−0.33, −0.09	−0.39	0.04	−9.02^***^	−0.48, −0.31	8.75^**^
RA on DS	−0.20	0.07	−3.01^**^	−0.33, −0.07	−0.40	0.04	−9.73^***^	−0.48, −0.32	7.93^**^

MHP, Mental health problems; LN, Loneliness; DS, Depressive symptoms; SE, Social equality; GR, Group responsibility; RA, Rule abiding. ^*^p < 0.05, ^**^p < 0.01, ^***^p < 0.001.

Finally, we further conducted multigroup analysis to test whether there were rural–urban group differences in the relations before to during the pandemic. The results of rural-group differences in the relations of group orientations on mental health problems before and during the pandemic are presented in Table 7. The Wald chi-square test indicated there were group differences between social equality [*χ*^2^(6) = 18.83, *p* < 0.01], group responsibility [*χ*^2^(2) = 7.72, *p* < 0.05, only constrained path coefficient of main effect] as well as rule abiding [*χ*^2^(6) = 18.31, *p* < 0.01] and mental health problems overall. Follow-up invariance tests indicated that before the pandemic, social equality, group responsibility and rule abiding were all negatively associated with loneliness and depressive symptoms in rural and urban, and no rural–urban group differences in the relations. However, during the pandemic, the associations of social equality, group responsibility and rule abiding on loneliness and depressive symptoms in urban, group responsibility on depressive symptoms in rural, were all significant, and there were rural–urban group differences [*χ*^2^(1) = 7.08 to 13.77, *p*s < 0.01] in the relations. In addition, the before-during pandemic group differences between social equality and loneliness [*χ*^2^(1) = 47.27, *p* < 0.001], rule abiding and loneliness [*χ*^2^(1) = 58.50, *p* < 0.001] and depressive symptoms [*χ*^2^(1) = 4.87, *p* < 0.05] were all significant in rural (rather than in urban).

**Table 7:** Rural-group differences in the relations of group orientations on mental health problems before and during the pandemic.

	Rural				Urban				
Path	*β*	*SE*	*t*	95%CI	*β*	*SE*	*t*	95%CI	*χ^2^*(1)
**SE on MHP**									
Bef: SE on LN	−0.43	0.13	−3.40^***^	−0.68, −0.18	−0.39	0.07	−5.82^***^	−0.53, −0.26	1.21
Dur: SE on LN	−0.10	0.08	−1.34	−0.25, 0.05	−0.35	0.06	−5.56^***^	−0.47, −0.23	12.63^***^
Bef: SE on DS	−0.37	0.13	−2.78^**^	−0.64, −0.11	−0.32	0.07	−4.97^***^	−0.45, −0.20	1.67
Dur: SE on DS	−0.09	0.09	−0.96	−0.26, 0.09	−0.36	0.06	−5.94^***^	−0.48, −0.24	8.71^**^
**GR on MHP**									
Bef: GR on LN	−0.35	0.10	−3.46^***^	−0.55, −0.15	−0.44	0.06	−6.77^***^	−0.56, −0.31	1.11
Dur: GR on LN	−0.22	0.08	−2.90^**^	−0.42, −0.07	−0.48	0.06	−7.47^***^	−0.60, −0.35	7.08^**^
Bef: GR on DS	−0.34	0.11	−3.13^**^	−0.56, −0.13	−0.36	0.06	−6.18^***^	−0.47, −0.24	0.89
Dur: GR on DS	−0.15	0.09	−1.74	−0.32, 0.02	−0.47	0.05	−8.85^***^	−0.57, −0.37	7.98^**^
**RA on MHP**									
Bef: RA on LN	−0.44	0.11	−3.86^***^	−0.66, −0.22	−0.41	0.06	−6.65^***^	−0.53, −0.29	0.28
Dur: RA on LN	−0.10	0.08	−1.32	−0.26, 0.05	−0.36	0.06	−5.82^***^	−0.49, −0.24	11.88^***^
Bef: RA on DS	−0.44	0.12	−3.63^***^	−0.67, −0.20	−0.36	0.06	−6.32^***^	−0.47, −0.25	0.07
Dur: RA on DS	−0.09	0.08	−1.07	−0.25, 0.07	−0.43	0.06	−7.21^***^	−0.54, −0.31	13.77^***^

Bef, Before the pandemic; Dur, During the pandemic; MHP, Mental health problems; LN, Loneliness; DS, Depressive symptoms; SE, Social equality; GR, Group responsibility; RA, Rule abiding. ^*^p < 0.05, ^**^p < 0.01, ^***^p < 0.001.

## 4. Discussion

By surveying rural and urban early adolescents shortly before and 2 years into the COVID-19 pandemic in China, we found that, compared with students before the pandemic, during-pandemic students displayed lower group orientation such as group responsibility and rule abiding of rural students, and increased loneliness and depressive symptoms. More importantly, we found stronger negative associations between group orientation and mental health problems in urban contexts than in rural ones. The protective effect of group orientation on mental health seems to weaken only in rural contexts. These results indicate different implications regarding group orientation and the mental health of urban and rural early adolescents facing threats posed by the COVID-19 pandemic in China.

We found that early adolescents’ loneliness and depressive symptoms were significantly higher during the pandemic than those before the pandemic. These results suggest that the pandemic has negatively impacted mental health, which could be explained by COVID-19-related restrictions (Liu et al., 2021). In line with previous studies (e.g., Chen et al., 2012), we found that girls reported higher group orientation, loneliness, and depressive symptoms than did boys.

Approximately 2 years after the COVID-19 outbreak, we found that both feelings of social equality and group responsibility decreased. These changes may be due to personal and societal disease prevention measures restricting behavior that expresses self-transcendence, such as altruistic behavior (e.g., helping classmates) and cooperation (e.g., actively negotiating conflict) during a continuous crisis event (Daniel et al., 2021). Alternatively, it is possible that concern for self-preservation and personal safety outweighs some concern for others, which is consistent with previous research suggesting that excessive worry may cause social withdrawal (Seligman, 1972). Contrary to previous hypotheses, we found that rule-abiding declined, and that group responsibility and rule-abiding were reduced only in rural students before and during the pandemic, not urban students. It may be that, although the tighter society-level preventive measures implemented in rural areas (e.g., closed access to villages and police-enforced social distancing) resulted in very low infection rates, the relatively wide living space and lack of disease knowledge rendered individual-level preventive measures (e.g., wearing facemasks and handwashing) difficult to monitor, leading to frequent violations of pandemic prevention measures, which may reduce rural adolescents’ acceptance of the values like group responsibility and rule-abiding. Moreover, as values can be transmitted intergenerationally (Knafo and Schwartz, 2004), the generally higher education level of urban adolescents’ parents may result in these teenagers receiving more attention, thus alleviating the decline of group orientation.

In line with earlier research findings (e.g., Li et al., 2018), we did not find a significantly stronger negative relationship between group orientation and mental health problems in rural areas. Further analysis revealed that the attenuating effect of each aspect of group orientation on mental health weakened or even disappeared in rural (but not urban) areas during the pandemic. This finding differs from those of previous studies (Chen et al., 2012; Liu et al., 2018). This may be related to new changes in external threat pressure over time. In the early stages of the COVID-19 pandemic, whether in urban or rural areas, the imposition of unfamiliar public health measures, infringements on personal freedoms, speculation about uncertain health prognoses, large and growing financial losses, conflicting and changing messaging from authorities, and severing of social connection contributed to widespread distress and risk of mental health difficulties (Pfefferbaum and North, 2020). Even rural migrant children and left-behind children appeared to have higher psychological well-being than urban children (Zhang R. et al., 2022). Approximately 2 years following the outbreak, however, while urban residents recovered quickly when virus transmission was effectively contained, the impact of the pandemic on rural regions remains unresolved, if not intensified (Shen et al., 2021). Persistent uncertainty and reduced sense of control make some rural adolescents less concerned about group interests, which is in line with research on learned helplessness (Seligman, 1972). Therefore, rural adolescents may benefit less from group orientation to prevent mental health problems than their urban peers.

In the specific context of the COVID-19 pandemic, previous studies had indicated that activating group orientation could promote prosocial behaviors among adolescents (e.g., Russo et al., 2022). It is also suggested by existential positive psychology and Wong et al.’s (2021) self-transcendence paradigm model that human beings can best flourish through the transformation of suffering and concern for others in a difficult and uncertain world. This study’s findings suggest the importance of social context in the relationship between value orientation and mental health symptoms. To create a good environment for cultivating adolescents value orientations during and after the pandemic, policymakers and educators should emphasize their growth and learning circumstances that minimize the influence of risk factors on adolescents’ values, especially in rural areas.

Several study limitations and future research directions should be noted. First, this study only identified changes in early adolescents’ group orientation and mental health during the pandemic, it did not elucidate how value orientations influence mental health. Future studies should examine the mechanisms through which group orientation affects loneliness, depressive symptoms, and other aspects of mental health, such as whether mental health problems can be alleviated through prosocial behaviors (Russo et al., 2022). Second, this research only focused on group orientation and did not address other, self-oriented values such as fashion and personal happiness. Previous studies have found that collectivistic and individualistic orientations coexist among young Chinese individuals (Tan et al., 2021). Third, the cross-sectional design, single-subject groups (Chinese ninth graders), and higher percentage of urban residents in the pre-pandemic sample prevents us from drawing causal conclusions and limits the generalizability of our findings. Finally, we examined societal changes in values using a self-report survey at the individual level, future research should use additional methods such as classify free-formatted texts according to the values that they express (Sagiv and Schwartz, 2022), and also encompass the cultural and social levels.

## 5. Conclusion

Overall, this study reveals that during a continuous crisis affecting many fields of life, environmental conditions may lead to change in the value orientation of early adolescents, with possible long-term implications for mental health. Two years after the outbreak of the pandemic, we found lower group orientation and more loneliness and depressive symptoms among early adolescents. Moreover, during the pandemic, the positive effects of group orientation on loneliness and depressive symptoms were stronger among urban adolescents than their rural peers. These results indicate that, during a continuous crisis event that affects many areas of life, value orientations and their relationships to mental health may change in multiple directions.

## Data availability statement

The raw data supporting the conclusions of this article will be made available by the authors, without undue reservation.

## Ethics statement

The studies involving human participants were reviewed and approved by Ethics Review Board of the Social Sciences Office of Shanghai Normal University. Written informed consent to participate in this study was provided by the participants’ legal guardian/next of kin.

## Author contributions

XH: conceptualization, methodology, formal analysis, resources, data curation, and writing—original draft. DL: conceptualization, methodology, writing—review and editing, and validation. MZ: data curation. YX, PY, XD, and RZ: methodology, investigation, and writing—review and editing. All authors contributed to the article and approved the submitted version.

## Funding

This study was supported by Key Innovation Project of Shanghai Municipal Education Commission (2019-01-07-00-02-E00005).

## Conflict of interest

The authors declare that they have no known competing financial interests or personal relationships that could appear to influence the work reported in this paper.

## Publisher’s note

All claims expressed in this article are solely those of the authors and do not necessarily represent those of their affiliated organizations, or those of the publisher, the editors and the reviewers. Any product that may be evaluated in this article, or claim that may be made by its manufacturer, is not guaranteed or endorsed by the publisher.
